# Case report: Coronavirus Disease 2019 (COVID-19) modified RNA vaccination-induced Adult-Onset Still's Disease with fulminant myocarditis as initial presentation

**DOI:** 10.3389/fcvm.2023.1066699

**Published:** 2023-03-15

**Authors:** Mi Zhou, Chun Ka Wong, Wan Yin Winnie Yeung, Chung Wah Siu, Lixue Yin

**Affiliations:** ^1^Cardiology Division, Department of Medicine, The University of Hong Kong, Hong Kong, Hong Kong SAR, China; ^2^Rheumatology Division, Department of Medicine, Queen Mary Hospital, Hong Kong, Hong Kong SAR, China; ^3^Cardiovascular Ultrasound and Non-Invasive Cardiology Department, Sichuan Provincial People's Hospital, Chengdu, China

**Keywords:** myocarditis, vaccine, mRNA vaccine, Adult-Onset Still's Disease (AOSD), autoimmune disease

## Abstract

Myocarditis is a rare complication of Coronavirus Disease 2019 (COVID-19) vaccination. We report a case of an elderly female who presented initially with acute myocarditis, fulminant heart failure, and atrial fibrillation after receiving a modified ribonucleic acid (mRNA) vaccine (BNT162b2). Unlike other patients with vaccine-induced myocarditis, she developed persistent fever, sore throat, polyarthralgia, diffuse macular rash, and lymphadenopathy. After extensive investigation, she was diagnosed with post-vaccination Adult-Onset Still's Disease. The systemic inflammation gradually subsided after the use of non-steroidal anti-inflammatory drugs and systemic steroids. She was discharged from hospital with stable hemodynamics. Methotrexate was subsequently given to maintain long-term remission.

## Introduction

The Coronavirus Disease 2019 (COVID-19) vaccine BNT162b2 was the first ever modified RNA-based (mRNA) vaccine that received U.S. Food and Drug Administration (FDA) approval for use. Despite the satisfactory safety profile in randomized controlled trials, mRNA vaccines were later shown to increase the risk of myocarditis in post-markerting surveillance studies (1). Hereby, we report an elderly female who developed myocarditis after BNT162b2 vaccination. Unlike most self-limiting myocarditis developed in patients after BNT162b2 vaccination, she suffered from fulminant heart failure and persistent systemic inflammatory responses with fever, polyarthralgia, and rash. She was eventually diagnosed with post-vaccination Adult-Onset Still's Disease (AOSD). Our case report highlights the features of AOSD and the process of diagnosing this rare but potentially lethal condition.

## Case presentation

A 72-year-old female with a history of hypertension, diabetes mellitus, hyperlipidemia, thyroidectomy, and osteoporosis developed a persistent fever in the week following the first dose of mRNA COVID-19 vaccine BNT162b2. Over the subsequent weeks, she developed progressive shortness of breath, sore throat, polyarthralgia, malaise, decreased appetite, and insomnia. She was given empirical antibiotics and non-steroidal anti-inflammatory drugs (NSAIDs) by another hospital, but her symptoms did not resolve (Table 1).

**Table 1:** Baseline clinical condition and timeline.

**Basic clinical information**	
Age, years	72
Sex	Female
Medical history	Hypertension, diabetes mellitus, hyperlipidemia, thyroidectomy, and osteoporosis
**Timeline (post-vaccination)**	
Week 1	Fever, sore throat, polyarthralgia, decreased appetite, malaise, and insomnia. Took acetaminophen
Week 2	Persistent fever and systemic symptoms. Progressive shortness of breath. Admitted to another hospital for management. Was given empirical antibiotics and non-steroidal anti-inflammatory drugs (NSAIDs). Symptoms persisted
Week 4	Transferred to our hospital for further management. On admission, body temperature 38.7°C, blood pressure 100/72 mmHg, heart rate 162 beats per minute, and oxygen saturation of 96% in room air. Electrocardiogram showed atrial fibrillation with rapid ventricular rate. Echocardiography showed impaired left ventricular ejection fraction 16–20%. Elevated troponin and brain natriuretic peptide found. Chest X-ray showed pulmonary congestion. Given diuretics to optimize fluid status, amiodarone for atrial fibrillation with rapid ventricular rate, and apixaban as anticoagulant. Subsequently developed shock requiring noradrenaline infusion and desaturation requiring high flow oxygen supplementation. Hemodynamic status improved after heart rate optimization
Week 5	Right coronary angiogram showed no obstructive coronary artery disease. Endomyocardial biopsy was not diagnostic of myocarditis. Cardiac magnetic resonance imaging established myocarditis diagnosis with modified Lake Louise criteria. All microbiological investigations were negative. Owing to persistent fever, polyarthralgia, and development of macular rash over trunk and limbs, initiated investigation for autoinflammatory syndromes
Week 7	Positron emission tomography (PET) showed lymphadenopathy over cervical, thoracic, and abdominal area with mildly raised hypermetabolic uptake signals. No infective foci or malignancy found
Week 8	After reviewing all investigations, diagnosis of Adult-Onset Still's Disease (AOSD) established. Initiated 30 mg prednisolone daily and 25 mg indomethacin three times per day. Fever and systemic symptoms gradually resolved
Week 14	Patient discharged from hospital after complete resolution of systemic inflammatory symptoms and rehabilitation. Echocardiography prior to discharge showed left ventricular ejection fraction (LVEF) of 57.5% and global longitudinal strain (GLS) of −17.5%. Segmental longitudinal strain of the anterior, anteroseptal, inferoseptal, and posterior walls at the basal and middle level remained decreased, as did the layer-specific strain from the epicardium to mid-myocardium
Week 54	Flare-up of AOSD with persistent low grade fever, sore throat, polyarthralgia, and rash. Started hydrocortisone and methotrexate. Discharged after resolution of symptoms
Week 60	Remained asymptomatic at latest follow up

She attended to the Accident and Emergency Department of our hospital 4 weeks after vaccination for the persistence of the aforementioned symptoms. Upon examination, she was found to have a fever with a body temperature of 38.7°C, blood pressure of 100/72 mmHg, heart rate of 162 beats per minute, and oxygen saturation of 96% in room air. Physical examination revealed bilateral basal crepitations but was otherwise unremarkable. Electrocardiogram (ECG) showed atrial fibrillation (AF) with a rapid ventricular response of 150–160 beats per minute with no ST segment or T wave change (Figure 1A). Troponin T peaked at 7,000 ng/ml and B-type natriuretic peptide (BNP) was grossly elevated to >26,000 pg/ml. She also had an elevated white blood cell count of 20.44 × 10^9^/L and a neutrophil count of 19.06 × 10^9^/L. C-reactive protein (CRP) was elevated at 22.4 ng/dL and the erythrocyte sedimentation rate (ESR) was raised at 28 mm/h. Liver parenchymal enzymes were raised with aspartate aminotransferase (AST) 112 U/L and alanine transaminase (ALT) 116 U/L (Tables 1, 2). Chest x-ray found pulmonary congestion. Thoracic computed tomography revealed no additional findings. Echocardiography found a left ventricular ejection fraction (LVEF) of 16–20% with global hypokinesia, moderate mitral regurgitation, and tricuspid regurgitation. There was no pericardial effusion.

**Figure 1:** Key investigations performed. **(A)** Electrocardiogram showing atrial fibrillation with rapid ventricular response. There was no significant ST segment or T wave change. **(B)** Coronary angiogram showed no obstructive coronar artery disease. **(C)** Positron emission tomography and computed tomography (PET-CT) showed lymphadenopathy over cervical, bilateral axillary, mediastinal, hilar, porta hepatis, and peripancreatic areas. **(D)** Cardiac strain analysis performed prior to discharge from hospital showed nearly normalized LVEF of 57.5% and global longitudinal strain (GL) of −17.5%. Decreased segmental longitudinal strain in anterior, anteroseptal, inferoseptal, and posterior from basal to mid level, and decrease in layer-specific strain from epicardial to mid-myocardial were observed.

**Table 2:** Investigations.

**Investigation**	**Result**
**Hematology**	
Hemoglobin, gm/dL	11.0
White blood cell, × 10^9^/L	20.44
Neutrophils, × 10^9^/L	19.06
Lymphocytes, × 10^9^/L	0.73
Platelets, × 10^9^/L	264
Prothrombin time, s	11.6
Activated partial thromboplastin time, s	28.8
**Biochemistry**	
Sodium, mmol/L	121
Potassium, mmol/L	2.7
Creatinine, mg/dL	40
Aspartate aminotransferase, U/L	112
Alanine transaminase, U/L	116
Total bilirubin, mg/dL	9
Alkaline phosphatase, U/L	136
Lactate dehydrogenase, U/L	1,424
**Inflammatory markers**	
Ferritin, pmol/L	68,913
Procalcitonin, ng/mL	1.2
Erythrocyte sedimentation rate, mm/h	28
C-reactive protein, ng/dL	22.4
**Cardiac biomarkers**	
Troponin T, ng/mL	7,000
Brain natriuretic peptide, pg/ml	> 26,000
**Microbiology**	
Nasopharynx and throat swab for viral nucleic acid PCR (influenza A and B virus, parainfluenza virus, severe acute respiratory virus type 2, enterovirus/rhinovirus, and respiratory syncytial virus)	Negative
Serology (enterovirus, hepatitis B and C, human immunodeficiency virus, rickettsia, scrub typhus, melioidosis, coxiella burnetiid, Epstein–Barr virus)	Negative
Plasma nucleic acid PCR (adenovirus)	Negative
Stool nucleic acid PCR (enterovirus)	Negative
Sputum, pleural fluid, and urine acid fast bacilli smear and culture	Negative
Sputum, pleural fluid, and urine mycobacterium tuberculosis PCR	Negative
Urine legionella antigen	Negative
Anti-Streptolysin-o, IU/ml	< 100
Cytomegalovirus PP65	Intermittent positive (mild)
**Autoimmune investigations**	
IgA, mg/dL	175
IgG, mg/dl	1,167
IgM, mg/dl	188
Anti-nuclear antibody, titer	1/80
Anti-double stranded DNA, IU/mL	1.2
Rheumatoid Factor, IU/mL	< 12
Anti-neutrophil cytoplasmic antibody	Atypical
Anti-extractable antigen, RNP	Negative
Anti-extractable antigen, Sm	Negative
Anti-extractable antigen, Ro	Positive
Anti-extractable antigen, La	Negative
Anti-proteinase 3, IU/mL	< 2.0
Anti-myeloperoxidase, concentration, pmol/L	7.6
Anti-glomerular basement membrane protein, %	< 1.5

PCR, polymerase chain reaction.

DCoronary angiography revealed no obstructive coronary artery disease (Figure 1B). An endomyocardial biopsy of the right ventricular septum was performed and histopathology was non-diagnostic. Cardiac magnetic resonance imaging was subsequently performed and found increased native relaxation time on T1 mapping and high signal intensity on T2 weighted mapping. Myocarditis was diagnosed according to the Lake Louise criteria (2). Microbiological investigations were arranged to rule out infective causes of myocarditis, including serology, nucleic acid detection by polymerase chain reaction, and culture in blood, urine, stool, throat swab, nasopharyngeal swab, and other body fluids (Table 2). After an extensive search, no infective foci were identified; she was labeled as having vaccination-induced myocarditis. She was given diuretics to optimize fluid status, amiodarone for atrial fibrillation with rapid ventricular rate, and apixaban for anticoagulation. Shortly after hospitalization, she developed an episode of shock requiring noradrenaline support and desaturation requiring high flow oxygen supplementation. Her hemodynamic conditions later stabilized when heat rate was adequately controlled.

Despite improvement in hemodynamic statutus, she was noted to have a persistent high fever, polyarthralgia, leukocytosis, and raised CRP. Ferritin was grossly elevated at 68,913 pmol/L. In addition, she was also noted to develop diffuse salmon pink non-itchy macular rash mainly over her trunk with some involvement of her limbs. Autoantibody screening, including antinuclear antibody, anti-double stranded DNA (anti-dsDNA), anti-extractable nuclear antigens (anti-ENA), and rheumatoid factor, were all negative (Table 2). Positron emission tomography and computed tomography (PET-CT) showed lymphadenopathy over cervical, bilateral axillary, mediastinal, hilar, porta hepatis, and peripancreatic areas with a maximum standard unit value (SUVmax) of 4.7. No malignancy, infective foci, or systemic feature of sarcoidosis was found (Figure 1C). Subsequent review by a multidisciplinary team including a cardiologist, hematologist, radiologist, and rheumatologist reached a diagnosis of AOSD based on the fulfillment of at least eight Yamaguchi criteria, including four major criteria, and after exclusion of infectious, malignant, and other autoimmune conditions (3) (Table 3). She was prescribed 30 mg of prednisolone daily and 25 mg of indomethacin three times per day. Her fever, rash, leukocytosis, and raised inflammatory markers gradually resolved. Transthoracic echocardiography and speckle tracking analysis performed prior to discharge found nearly normalized LVEF of 57.5% and global longitudinal strain (GLS) of −17.5%. Segmental longitudinal strain of the anterior, anteroseptal, inferoseptal, and posterior walls at the basal and middle level remained decreased, as did the layer-specific strain from the epicardium to mid-myocardium (Figure 1D). She was discharged from hospital after a prolonged course of rehabilitation and in-patient monitoring at 14 weeks post-vaccination.

**Table 3:** Diagnostic considerations.

**Yamaguchi criteria for Adult-Onset Still's disease**	
**Major criteria**	**4 out of 4**
Fever 39°C lasting ≥1 week	Present
Arthalgia or arthritis lasting ≥2 weeks	Present
Typical non-pruritic salmon-colored rash	Present
Leukocytosis ≥10,000/mm^3^ with granulocytes 80%	Present
**Minor criteria**	**4 out of 5**
Sore throat	Present
Lymphadenopathy	Present
Splenomegaly	Absent
Abnormal liver function test	Present
Negative tests for antinuclear antibody and rheumatic factor	Present
**Exclusion criteria**	**0 out of 3**
Infection	Excluded
Malignancy	Excluded
Other rheumatic disease	Excluded
**Major differential diagnosis excluded**	
**Infective myocarditis:** Excluded by extensive microbiological investigations	
**Sarcoidosis:** Rarely present in Chinese ethnicity. No evidence of systemic sarcoidosis on positron emission tomography and computed tomography (PET-CT).	
**Myocardial infarction:** No obstructive coronary artery disease on catheter-based coronary angiogram.	

At 9 months post-vaccination, our patient was again admitted with a flare-up of AOSD. She presented with persistent low-grade fever, sore throat, polyarthalgia, and macular rash most apparent over the ankles, upper limbs, and buttock region. She was prescribed hydrocortisone and methotrexate after excluding any infectious cause. Her symptoms gradually resolved and she remained asymptomatic as of time of this writing. Serial echocardiography will be arranged for this patient in subsequent follow-up to monitor changes of the currently impaired segmental longitudinal strain.

## Discussion

The recently approved mRNA vaccines for COVID-19 have generally shown an outstanding safety profile. However, in a minority of cases, new onset or flare-up of autoimmune diseases may develop after COVID-19 vaccination. The precise mechanism underlying these autoimmune phenomena is currently unknown, with various postulations including molecular mimicry and cytokine surges leading to a systemic inflammatory state and more (4, 5). Myocarditis is one of the most concerning complications associated with mRNA vaccination as it is potentially lethal (1). Our patient presented with a fulminant systemic inflammatory response with AOSD complicated with myocarditis and heart failure. Establishing the diagnosis of AOSD with the initial presentation being myocarditis was challenging. After appropriate anti-inflammatory therapies, her hemodynamic condition improved and systemic inflammation resolved.

AOSD is a rare autoinflammatory disease characterized by persistent fever, rash, polyarthralgia, sore throat, leukocytosis, neutrophilia, lymphadenopathy, hepatomegaly, splenomegaly, and abnormal liver function (6). AOSD is classified according to the Yamaguchi criteria (3), which requires the fulfillment of five or more criteria with two being major criteria (Table 3). The main criteria include fever ≥39°C for ≥1 week, arthralgia or arthritis for ≥2 weeks, typical non-pruritic salmon-colored rash, and leukocytosis ≥10,000 /mL with ≥80% granulocytes. The minor criteria include sore throat, lymphadenopathy, splnomegaly, abnormal liver function, and negative antinuclear antibody and rheumatoid factors. The exclusion of infection, other autoimmune disesases, and neoplasm are also required. In terms of cardiac manifestation, AOSD patients may develop pericarditis and myocarditis. In rare case reports, new onset severe mitral regurgitation was also suggested to be related to AOSD (7). Although AOSD following mRNA vaccines is rare (8–10), it is critical for clinicians to be knowledgable about the condition as it is potentially life threatening, as in our patient who developed systemic inflammatory response and unstable hemodynamics from arrhythmia and heart failure. Prompt initiation of anti-inflammatory agents is mandatory to avert clinical deterioration and mortality.

## Conclusion

AOSD with fulminant myocarditis is a rare but potentially life-threatening complication of COVID-19 mRNA vaccines. It is critical to promptly establish the correct diagnosis and initiate anti-inflammatory therapy to avert clinical deterioration and mortality.

## Data availability statement

The original contributions presented in the study are included in the article/supplementary material, further inquiries can be directed to the corresponding authors.

## Ethics statement

The study protocol was approved by the Institutional Review Board of the University of Hong Kong and Hong Kong West Cluster, Hospital Authority of Hong Kong (UW21-214). Written informed consent was obtained from the patient for publication of any potentially identifiable images or data included in this article.

## Author contributions

MZ, CWS, and LY conceived and designed the study. MZ wrote the first draft of the manuscript. CKW, WYWY, and CWS performed critical revision of the manuscript. All authors contributed to the article and approved the submitted version.
